The article "The usage of spatial econometric approach to explore the determinants of ecological footprint in BRI countries" was retracted in 2024. Reasons: compromised peer review; unreliable results or conclusions; concerns about the data; concerns about the peer review.

# The usage of spatial econometric approach to explore the determinants of ecological footprint in BRI countries

**DOI:** 10.1371/journal.pone.0288683

**Published:** 2023-10-31

**Authors:** Qian Chen, Ghulam Rasool Madni, Adnan Ali Shahzad

**Affiliations:** 1 Law School of Shanghai University of Finance and Economics, Shanghai, 200433, China; 2 Department of Economics, Division of Management and Administrative Science, University of Education, Lahore, Pakistan; Hamdard University, PAKISTAN

## Abstract

Protecting our environment is not a choice, but a responsibility we owe to future generations. Numerous studies examined the factors affecting the environmental deterioration but this research takes a step further by employing a spatial dependence model to evaluate spatial impact of ecological footprint and its contributing factors, particularly productive capacities which is hardly investigated in economic literature of BRI economies. For the purpose, the annual data of 54 BRI countries is analyzed for the time period from 2000 to 2018 by employing various econometric techniques. The outcomes of the Durbin model express that neighboring economies significantly affect the ecological footprint of an economy, highlighting the need for a regional policy framework to address environmental issues. It is also found that improving the productive capacities, green investment and democratic quality decrease the ecological footprint while per capita GDP, globalization, and development of financial sector increase the environmental deterioration. The significant interdependence of the countries within the region, a regional policy and vision must be implemented to safeguard the environment. The research findings can facilitate policy formulation aimed at promoting environmental sustainability, with particular focus on enhancing productive capacities and green investments.

## 1. Introduction

The rising GHG emissions and associated climatic changes are presently worldwide challenges [1]. It is estimated thatchange1.5 centigrade global temperature has been increased after industrial revolutions [2]. Due to rapid industrial expansion, the natural resources and environmental sustainability are on threat [3]. The global economies are struggling hard to offset the degradation of environment as a result of economic expansion. On the one side, countries are trying hard to improve the living standard through growth. On the other side, there is huge consumption of natural resources on behalf of rapid economic expansion resulting biodiversity loss, degradation of land, pollution, and exploitation of resources [4–6]. The fundamental goal is to achieve the higher levels of growth while maintaining the environmental quality by establishing a balance between human needs and the earth’s natural inherent ability for regeneration of resources. Countries are making efforts to slow the process of environmental deterioration [7–12].

The article "The usage of spatial econometric approach to explore the determinants of ecological footprint in BRI countries" was retracted in 2024. Reasons: compromised peer review; unreliable results or conclusions; concerns about the data; concerns about the peer review.

The comprehensive indicator to measure the environmental degradation is ecological footprint while its spatial impact is hardly discussed in the earlier literature [13]. The spatial impact of ecological footprint refers to the assessment of how ecological footprints vary and are distributed across different regions or areas [14]. This analysis helps to identify the regions with high environmental impact, understand the factors driving environmental degradation in specific areas and uncover interconnectedness among regions [15]. There are several reasons to determine the spatial impact of ecological footprint. Firstly, understanding the spatial distribution and variation of ecological footprints allows us to identify regions or areas that are experiencing higher levels of environmental impact [16]. This information helps us to prioritize the areas that require immediate attention in terms of environmental management. Secondly, we are able to uncover the underlying factors and drivers that contribute to environmental degradation in specific regions [17]. This knowledge enables policymakers and stakeholders to design effective strategies and interventions to mitigate negative environmental impacts and promote sustainable practices. Furthermore, examining the spatial patterns of ecological footprints can reveal the interconnectedness and interdependencies among different regions [18]. It allows us to understand how environmental pressures and resource consumption in one area may affect neighboring or distant regions through environmental flows, such as air pollution, water contamination, or ecosystem degradation. This holistic understanding of spatial interactions provides a basis for developing collaborative approaches and transboundary initiatives to address environmental challenges collectively.

If we have a look on potential determinants to affect the ecological footprint in a country or region then numerous factors are found in literature like green investment, globalization, per capita GDP, financial development, democratic quality [19–23] but role of productive capacities is hardly discussed in earlier studies. Productive capacities refer to an economy’s ability to produce goods and services using its available resources, such as labor, capital, and technology. It can be measured in terms of a country’s level of industrialization, technological advancement, and workforce skills [14]. A country with high productive capacities is able to efficiently utilize its resources, increase its output, and compete more effectively in the global market. The United Nations constructed the “Product Capacities Index” (PCI) [18], which highlights the comprehensive productive structure of a country.

The article "The usage of spatial econometric approach to explore the determinants of ecological footprint in BRI countries" was retracted in 2024. Reasons: compromised peer review; unreliable results or conclusions; concerns about the data; concerns about the peer review.

There are many solid motivations for doing this study for BRI economies. Firstly, it covers a wide range of geographic area along with almost half global population and diverse economies as the Chinese report highlights that “65 countries will actively engage in the BRI, including 24 from Europe, 15 from North Africa and the Middle East, and 26 from Asia, 30% of the world’s GDP and 4.4 billion people are involved in this venture. In addition to these 65, 48 more countries have expressed their desire to actively engage in the BRI project” [13]. Moreover, there are serious environmental concerns due to this project because energy consumption has significantly increased as a result of modernization of industrial sector of the BRI countries. From the beginning to 2019, “China invested US$760 billion, of which 39% went to the energy sector because BRI nations are generating 74.69% of the world’s coal, 53.82% of its natural gas, and 55.17 percent of its known crude oil reserves” [24]. These traditional sources of energy are responsible for 28% of CO2 emission and expected to increase by 66% till 2050 [25]. The BRI economies are particularly vulnerable to environmental problems due to their heavy reliance on natural resources [25]. It is important to study the spatial impact of ecological footprint and to identify the determinants of ecological footprint in BRI countries to understand the factors contributing to environmental degradation and to develop policies and strategies to mitigate its negative impacts.

This investigation differs from past studies in a few respects. This paper investigates the spatial impact of ecological footprint and its determinants for 54 BRI member economies covering the time period of 2000–2018. The spatial econometric approach is applied to determine the spatial dependence of ecological footprint. It will be helpful to understand the impact of environmental performance of a country on environmental conditions of neighboring countries. The research’s novelty lies in comprehensive and quantitative analysis of spatial perspective of ecological footprint in context of BRI countries specifically, contributing to the advancement of knowledge in understanding and addressing environmental challenges in the region. Moreover, by providing insights into the relationship between productive capacities and ecological footprint, it aids in formulating effective policies, advancing sustainable development goals, and fostering awareness about ecological footprints. It highlights the need to assess the spatial distribution of ecological footprints to identify areas of high environmental stress and inform targeted mitigation measures. By analyzing the spatial impact of ecological footprints, policymakers can identify regions that require specific attention for environmental conservation, resource management, and sustainable development initiatives.

The article "The usage of spatial econometric approach to explore the determinants of ecological footprint in BRI countries" was retracted in 2024. Reasons: compromised peer review; unreliable results or conclusions; concerns about the data; concerns about the peer review.

## 2. Theoretical foundations and earlier literature

The primary objectives of this study are explorations of spatial impact and potential factors of ecological footprint. In this section, the theoretical relationship of potential determinants affecting the ecological footprint, is established. These determinants include productive capacities, green investment, democratic quality, per capita GDP, globalization and financial development. It is worth noting that impact of productive capacities on ecological footprint is hardly explored in the literature so this research is a pioneering study to open the debate. The productive capacities are measured through “productive capacities index” that is made up of eight major components with 46 sub-indicators, such as “information and communication technology (ICT), structural change, natural capital, human capital, energy, transport, the private sector, and institutions” [18]. It may be argued that PCI is the most comprehensive and in-depth measure ever identified to assess productivity of a country. High PCI values indicate a productive economic structure for a nation, whereas lower PCI levels indicate a less productive economy. Through several paths, each indicator of productive capacity index has a link with environmental quality. The relationship of each indicator with environment is mentioned below.

“Information and communication technology” (ICT), is a key element of PCI. It encompasses the extent to which the internet, telephones, and mobile phones are used [26]. ICT has the potential to affect the environment as well because it increases productivity, reduces energy use, and hence reduces CO2 emissions [27,28]. The structural change in economy is another important component in deciding whether environmental quality is improving or falling. As the economy shifts from agriculture to industry, the demand for energy rises. [29]. Natural capital is crucial for both productivity and sustained economic development [30]. Natural resources may have an impact on the environment. Numerous studies have shown that productivity increases due to human capital and it has a direct and indirect impact on growth [31,32]. Equitable and long-term growth are seen to depend critically on energy performance [33]. Energy consumption will decrease as energy efficiency increases, reducing the harm to the environment. An important component of ensuring energy efficiency is transportation convenience. Investment in transport sector encourage economic growth by saving time and money and sharply increasing regional productivity [34]. This improvement results in less energy being used and less pollutants being created. Given that the transport sector is responsible for about 18% of the world’s CO_2_ emission, this is highly significant. On the one hand, transportation increases output, but its reliance on fossil fuels also increases the risk of greater degradation [35]. The private sector promotes productivity through generating jobs for citizens, providing goods and services, increasing tax revenue for the government, and making a large contribution to the development of technology [36,37]. The expanding role of the private sector may be advantageous for the environment by using eco-friendly technology [38]. Studies have shown that inadequate institutional quality hinders the productive potential of developing economies and serves as a barrier for environmental preservation [39]. Improving the institutional quality can dramatically reduce CO2 emissions while increasing production with the use of monitoring and regulatory rules [40].

The article "The usage of spatial econometric approach to explore the determinants of ecological footprint in BRI countries" was retracted in 2024. Reasons: compromised peer review; unreliable results or conclusions; concerns about the data; concerns about the peer review.

Green investment has a significant impact on ecological footprint in BRI countries [20]. Green investment is considered as an investment in sustainable technologies and practices that reduce environmental deterioration and promotion of sustainable development. These investments can lead to reduced CO2 emissions and increased use of renewable energy [21]. The literature highlights that green investment leads to reduction in the ecological footprint in BRI countries by promoting sustainable economic growth because green investment help to create more efficient and sustainable production process, reduce waste and pollution, and promote the use of renewable energy [18]. Overall, green investment is a crucial tool in promoting sustainable development and reducing the ecological footprint in BRI countries. Governments and businesses can work together to promote and invest in sustainable technologies and practices that can lead to a more sustainable future. The report of 2020 by the UN Industrial Development, “the energy consumption in transitional and emerging nations would increase by 50% over the next 25 years, growing from 1.8 to 3.1 in the industrial sector”. The summary of some other studies are reported in Table 1.

**Table 1:** Studies explaining factors of environmental deterioration.

Author/s	Environmental Variable	Territory	Methodology	Determinants of Environmental Deterioration
Pata [4]	CO2	USA	EKC Hypothesis	Globalization, Economic Complexity, Renewable Energy
Langnel & Amegavi [5]	Ecological Footprint	Ghana	ARDL	Globalization, Electricity Consumption
Saud et al. [9]	Ecological Footprint	BRI countries	PMG	Financial Development, Globalization
Shahbaz et al. [6]	CO2	India	ARDL	Energy consumption, globalization, financial development
Kamal et al [10]	CO2	105 countries	FMOLS	Fiscal policy, Trade openness, financial development, population
Charfeddine	Ecological	Qatar	Markov	Energy consumption,
[7]	Footprint, CO2		switching equilibrium correction model	Economic development
Chen & Madni [13]	Ecological Footprint	BRI countries	Driscol Kraay Method	Natural Resources, Green Investment, Globalization
Apergis et al. [14]	CO2	High Income countries	ARDL	Exports
Dogan et al [17]	CO2	55 countries	Panel quantile regression	Economic complexity, Urbanization, Energy consumption, Trade Openness
Chatti [27]	CO2	43 Countries	GMM	ICT, Transportation
Nathaniel & Khan [11]	Ecological Footprint	ASEAN	STIRPAT	urbanization, trade, renewable energy
Wang et al [28]	CO2	UK	Rolling Forecast	ICT

The democratic quality of a country has been found to have an impact on ecological footprint [13]. A higher level of democratic quality is associated with a lower ecological footprint, suggesting that democratic countries tend to be more environmentally conscious and prioritize sustainable development. This may be due to the greater public participation in decision- making processes and the presence of stronger institutions that promote environmental protection [9]. On the other hand, countries with lower democratic quality may prioritize economic growth over environmental protection, leading to a higher ecological footprint [14]. Therefore, promoting democratic values and institutions can ensure environmental preservation and sustainable development.

The article "The usage of spatial econometric approach to explore the determinants of ecological footprint in BRI countries" was retracted in 2024. Reasons: compromised peer review; unreliable results or conclusions; concerns about the data; concerns about the peer review.

In concluding, numerous studies explored the factors playing their role to deteriorate the environment but there is hardly any study which explored the impact of productive capacities on ecological footprint in the BRI region. It allows for effective environmental management, promotes sustainable practices, and helps in achieving long-term environmental sustainability. Moreover, being the importance to determine the spatial impact of ecological footprint, literature has an ample space to be filled by the further research. This study is an effort to fill this gap by determining the impact of productive capacities on ecological footprint and its spatial impact. It will help the policy makers, concerned authorities and researchers for targeted conservation efforts, efficient resource allocation, identifying vulnerable areas, advancing scientific knowledge, informing policy and decision-making process.

## 3. Methodology

### 3.1. Data and its sources

The annual panel data of 54 BRI economies is considered for empirical investigation covering the time span of 2000–2018. The sample is selected subject to data availability while data sources are Global Footprint Network, World Development Indicators, and Freedom House.

The environmental deterioration due to economic activities is measured through ecological footprint [41]. It has the capacity to track how human actions affect the environment. Environmental destruction increases as ecological footprint increases [42–44]. On the basis of earlier literature, it is hypothesized that per capita GDP, globalization, productive capacities, green investment, democratic quality and financial development are potential factors affecting the ecological footprint in the BRI economies. The description of data is given in Table 2.

**Table 2:** Description of data.

Variable	Symbol	Measurement	Sources
Ecological Footprint	ECF	Global Hectare	Global footprint network
Per Capital GDP	GDP		WDI
Globalization	GLB	KOF Index	KOF Swiss Economic Institute
Financial Development	FND	Index	WDI
Productive Capacities	PCP	Index	UNCTAD
Green Investment	GRI	Public Investment in Renewable Energy	International Renewable Energy Agency
Democratic Quality	DQL	Index	Freedom House

An index of democratic quality is constructed by taking aggregate values of civil liberty index and political rights index. These indices are built by Freedom House by taking into account multiple sub indicators representing different groups of statements like independence of judiciary, free media and press, rule of law, democracy, public voice, and individual rights. In the same way, the “civil liberty index” is built on 15 freedom relevant questions showing the individuals liberty in a territory. These two indices are combined by following the methodology developed by Charfeddine and Mrabet [45]. As the index adopts higher value, it represents the higher level of democracy and greater civil freedom. The principal component analysis is applied to construct the financial development index (FDI) as proposed by Nathaniel et al. [46]. If we want to simplify and reduce the dimensions of multivariate data, then PCA is an efficient statistical tool to handle such type of data and it is often used in environmental studies. The huge number of variables are transformed into few new variables and these new variables are labeled as principal components [47]. The FDI is built by joining the variables of domestic credit to private sector, foreign direct investment, and domestic credit to the private sector by banks. All the variables of FDI are measured as percentage of GDP.

The article "The usage of spatial econometric approach to explore the determinants of ecological footprint in BRI countries" was retracted in 2024. Reasons: compromised peer review; unreliable results or conclusions; concerns about the data; concerns about the peer review.

### 3.2. Model

The spatial dependence model may be employed to determine the spatial dependence of ecological footprint [48]. Spatial Dependence Model has several advantages as it accounts for the spatial effects that are commonly present in spatial data. This is particularly useful in situations where the data exhibit spatial autocorrelation or spatial heterogeneity. By accounting for spatial effects, the Spatial Dependence Model can lead to a better model fit, especially when compared to traditional regression models that ignore spatial dependence. The Spatial Dependence Model is robust to the presence of outliers and can handle non-normal errors. Moreover, it can help identify policy- relevant variables that influence the spatial distribution of the dependent variable and it can lead to better predictions of the dependent variable in unsampled areas by incorporating the spatial autocorrelation in the model. Spatial dependence reveals the spatial correlation among independent measured values in a specific geographical area. It explains the effects of a unit occurred due to actions in other units. It is used to determine the geographical relevance of an attribute between a spatial unit and neighboring spatial unit. The magnitude of spatial dependence is measured through Moran’s I value. Global Moran’s I value describe the correlation of ecological footprint across the sample area. The correct model specification and existence of spatial auto-correlation are determined through “Global Moran’s (GM’s) I test” [49]. The “GM’s I” test is specified as:

$$I=\frac{n\sum_{i=1}^{n}\sum_{j=1}^{n}Wij(\mathrm{Yi}‐\bar{Y})(\mathrm{Yj}‐Y)}{\sum_{i=1}^{n}\sum_{j=1}^{n}Wij\sum_{i=1}^{n}{\left(Yi-Y\right)}^{2}}$$ (i)

The n in the above specification shows the number of economies while Yi and Yj denote the ecological footprint of economy *i* and *j*. Wij represents the spatial weight matrix (SWM). GM’s I describes the spatial auto correlation index. It measures the spatial association among units through adding information of spatial relationship. The spatial matrix is built when it is judged for all adjacent relationship. Rook contiguity, k-nearest neighbors, and queen contiguity are few algorithms used to judge the adjacent relationships. The presence of adjacent relationship is considered by k-nearest neighbors and rook contiguity judges the edge adjacent, while corner adjacency is added by queen contiguity on the basis of rook contiguity. The rook contiguity is used for construction of row standardized SWM. The value of GM’s I test lies between -1 to 1. The value near to 1 reveals the strong positive spatial correlation while value closer to -1 highlights the strong negative spatial correlation. The positive spatial correlation is interpreted if the test statistics have the value more than 0 while value below than zero is considered as negative spatial correlation. No spatial correlation exists if the value is equal to zero [50]. The Z value is applied to find the significance level of GM’s I test following the standard normal distribution. The derivation is as follows:

$$Z_{I}=\frac{I-E[I]}{\sqrt{}\mathrm{Var}[I]}$$ (ii)

In above equation, E[I] is expected value while Var [I] shows the variance of GM’s I.

The article "The usage of spatial econometric approach to explore the determinants of ecological footprint in BRI countries" was retracted in 2024. Reasons: compromised peer review; unreliable results or conclusions; concerns about the data; concerns about the peer review.

The “spatial autocorrelation model” (SAC), “spatial error model” (SEM), and “spatial autoregressive model” (SAR) are different categories of spatial econometrics model. The SAC model shows the spatial dependence between error term and dependent variable. The specification of SAC model is as follows;

$$z=\alpha W_{1}z+\beta i_{n}+ϒB+\mu$$ (iii)

where μ shows autoregressive behavior and is equal to ηW2μ + ϵ while W1 matrix is considered equal to W2.

The spatial dependence of error term is determined through SEM model and specification of SEM model is as follows;

$$z=\beta i_{n}+ϒB+\mu$$ (iv)

while μ = ηWμ + ϵ where η shows the autoregressive behavior.

The spatial dependence in explained variable is determined through SAR model. The matrix from of SAR model is represented as:

$$z=\alpha Wz+\beta i_{n}+ϒB+\epsilon$$ (v)

The z in above equation represents the vector of n*1 observation for each unit of endogenous variable, W is a matrix of spatial weights, *i*n shows the vector of ones, B is a matrix of regressors, k denotes the number of regressors while α and β are coefficients, ϒ represents the vector of parameters, and ϵ shows error term.

The spatial dependence of lagged values of independent and dependent variables are estimated through “spatial Durbin model” (SDM) and specification of SDM is given as follows;

$$z=\alpha Wz+\beta i_{n}+ϒB+\varphi WB+\epsilon$$ (vi)

These four types of spatial models are regressed to find the spatial dependence and the findings of that model are selected which showed highest goodness of fitness. The SDM model has the ability to combine both SEM and SAR models so strategy of Belotti et al. [51] and LeSage and Pace [49] is adopted. We started with SDM to exclude the variables using likelihood ratios. The econometric model for estimation is as following:

$$ECF=a+\alpha WECF+{ϒ}_{1}GDP+{ϒ}_{2}GLB+{ϒ}_{3}FND+{ϒ}_{4}PCP+{ϒ}_{5}GRI+{ϒ}_{6}DQL+\varphi_{1}WGDP+\varphi_{2}WGLB+\varphi_{3}WFND+\varphi_{4}WPCP+\varphi_{5}WGRI+\varphi_{6}DQL+\epsilon$$ (vii)

where ECF is ecological footprint and represents the dependent variable as a proxy of environmental deterioration, while exogenous variables are per capita GDP, GLB (globalization), FND (financial development), PCP (production capacities), GRI (green investment), and DQL (democratic quality).

The article "The usage of spatial econometric approach to explore the determinants of ecological footprint in BRI countries" was retracted in 2024. Reasons: compromised peer review; unreliable results or conclusions; concerns about the data; concerns about the peer review.

## 4. Empirical findings

The Table 3 incorporates the empirical findings of GM’s I index. The Z values are highly significant and positive, revealing the spatial dependence of ecological footprint. So we can perceive the superiority of spatial model as compared with classic model.

**Table 3:** GM’s I index for dependent variable.

Years	2000	2001	2002	2003	2004	2005	2006	2007	2008	2009
GM’s I	0.351	0.313	0.372	0.411	0.427	0.284	0.394	0.363	0.418	0.438
p value	0.001	0.002	0.001	0.003	0.001	0.001	0.002	0.001	0.003	0.001
z value	3.684	4.258	4.511	4.387	4.361	3.995	3.867	4.027	5.177	4.337
**Years**	**2010**	**2011**	**2012**	**2013**	**2014**	**2015**	**2016**	**2017**	**2018**	
GM’s I	0.391	0.424	0.457	0.321	0.284	0.219	0.374	0.425	0.433	
p value	0.002	0.001	0.003	0.004	0.001	0.000	0.002	0.000	0.001	
z value	4.667	4.381	4.628	5.271	4.379	5.391	4.392	3.628	4.582	

The outcomes of the regression are pasted in the Table 4. It is revealed that SDM is an excellent model to reveal the impacts of exogenous variables on ecological footprint on the basis of highest value of adjusted R^2^ and lowest values of HQ, SC, and AIC. To determine the stability of empirical outcomes, four spatial models are regressed by employing “spatial weight matrices”, in addition of “Queen based contiguity weight matrix”, “K nearest contiguity weights matrix”, and “double rook contiguity weight matrix”. The LR test and goodness of fitness also declare the superiority of SDM as compared with other spatial models. The findings of selected spatial weight matrix are reported in the Table 4.

**Table 4:** Spatial models.

Variables	SEM	SAR	SAC	SDM
GDP	0.468*(0.019)	0.378*(0.011)	0.417* (0.019)	0.467*(0.010)
GLB	0.049 (0.052)	0.043 (0.072)	0.051 (0.052)	0.087***(0.042)
FND	0.212**(0.025)	0.243***(0.019)	0.222**(0.0211)	0.213*(0.0198)
PCP	-0.337**(0.086)	-0.044**(0.088)	-0.325**(0.099)	-0.295**(0.092)
GRI	-0.025* (0.004)	-0.028*(0.003)	-0.020* (0.003)	-0.029* (0.005)
DQL	-0.042*(0.004)	-0.051*(0.003)	-0.044*(0.004)	-0.049*(0.002)
Constant	-1.952**(0.318)	-2.998**(0.411)	-3.261**(0.284)	-4.974**(0.841)
**Spatial Effect**				
α		0.058(0.051)	0.071(0.049)	0.193(0.081)
φ	0.473**(0.071)		0.498**(0.070)	
W*GDP				-0.542*(0.039)
W*GLB				-0.087(0.991)
W*FND				-0.982***(0.059)
W*PCP				-0.885*(0.025)
W*GRI				-0.032**(0.016)
W*DQL				0.021**(0.195)
**Model Fitness**				
F-statistics	583.462**	674.664*	588.367*	619.528*
p-value (F-statistics)	0.003	0.005	0.004	0.003
R2	0.921	0.935	0.918	0.966
Adjusted R^2^	0.911	0.914	0.901	0.952
HQ	0.0528	0.427	0.512	0.384
SC	0.0589	0.557	0.618	0.332
AIC	0.0518	0.426	0.551	0.365

Note: *,**, and *** show significance level at 1%, 5% and 10% respectively in numerical figures. The empirical findings of spatial Durbin model depict that lagged endogenous variable has a positive relationship. The estimated value conveys that one-unit increase in ecological footprint of neighboring countries increases the ecological footprint in own state by 0.193 unit. Moreover, remaining spatial lagged exogenous variables have a significant relationship except for W*GLB and W*DQL.

The article "The usage of spatial econometric approach to explore the determinants of ecological footprint in BRI countries" was retracted in 2024. Reasons: compromised peer review; unreliable results or conclusions; concerns about the data; concerns about the peer review.

There are several robustness tests that can be performed to assess the validity and reliability of a Durbin spatial dependence model like Moran’s I Test which assesses whether the residuals of the model show spatial autocorrelation. If the residuals are spatially autocorrelated, it suggests that the model may not have fully captured the spatial dependence in the data. Lagrange Multiplier (LM) Test helps to identify whether there is any omitted variable bias in the model. It examines the null hypothesis that there is no spatial dependence in the model, and if the test rejects the null hypothesis, it suggests that the model suffers from omitted variable bias. Variance Inflation Factor (VIF) test is used to identify the presence of multicollinearity among the independent variables. If the VIF values are high, it suggests that there is a high degree of correlation between the independent variables, which can cause problems in estimating the model coefficients. Cross- Validation test involves dividing the data into training and testing sets to evaluate the model’s predictive power. If the model performs well in predicting the values in the testing set, it suggests that the model is robust and reliable.

## 5. Discussion

As it is assumed, the ecological footprint is highly impacted by per capita GDP. According to predicted values, a unit increase in per capita GDP increases the ecological footprint of 0.467 unit. This outcome is consistent with numerous earlier studies [41,46], which show that environmental quality deteriorates as per capita income rises because it increases the human demand on natural resources. A rise in income level of a bordering nation result in a large reduction in ECF of the home country as conveyed by “spatially lagged income variable” (W*GDP), which also has a significant and negative effect on the ecological footprint. Li and Li’s [52] investigation on the factors influencing carbon emissions in China supports these findings. It can be argued that economic activities expand when income level of country rises so production increases which deteriorates the environment.

The article "The usage of spatial econometric approach to explore the determinants of ecological footprint in BRI countries" was retracted in 2024. Reasons: compromised peer review; unreliable results or conclusions; concerns about the data; concerns about the peer review.

The empirical findings show that green investment and its spatially lag variable (W*GRI) have negative relationship with dependent variable, demonstrate that shifting from traditional ways to modern ways of production improve the quality of environment in home and neighboring countries. Despite the huge potential of renewable energies, Kahia et al. [53] and Nathaniel et al. [46] observed that the area has been experiencing severe environmental issues brought on by the widespread usage of fossil fuels. Fossil fuel use in BRI economies can result in air pollution that travels across borders and degrades the environment in nearby nations. The investment in pro- environment technologies and techniques save the environment even economic activities are expanded.

According to the coefficient of globalization, which is positive and significant, an increase in a country’s trade flow by one unit leads to increase its ECF by 0.087 unit. Since fossil fuels account for a significant portion in production sector of BRI participating countries, and these fossil fuels harm the environment so globalization is deteriorating the environment in case of BRI countries. A massive literature on the topic [14,15] have supported the findings of this study. However, there are several researches that disagree with our conclusions. For instance, it has been discovered that globalization can raise quality of environment due to transfer of cleaner technologies from industrialized nations through international commerce, which can lower ecological consumption [29,30]. The spatially lagged variable of globalization is not significant statistically.

The relationship between productive capacities and ecological footprint is negative, and spatial lagged coefficient (W*PCP) has a significant and negative relationship. It shows that productive capacities have capability to improve the environment of a country and it also improves the quality of environment in neighboring country. Because productive capacities are associated with improved living standard, easy access to cleaner technology, and higher demand for neat and clean environment. Productive capacities emphasize on information and communication technology, structural change, human capital, and social capital. So as potential of productive capacities increases, people demand rules and regulations to protect the environment for future generations. These findings are also backed up by Liu & Sagan [50] regarding their findings on CO2 emission in China.

The article "The usage of spatial econometric approach to explore the determinants of ecological footprint in BRI countries" was retracted in 2024. Reasons: compromised peer review; unreliable results or conclusions; concerns about the data; concerns about the peer review.

It is also worth noting that democratic quality is helpful to improve and sustain the environment. These outcomes are consistent with findings of You et al. [54] for 41 BRI economies, Haldar and Sethi [55] for 39 developing economies, and Al-Mulali and Ozturk [42] for MENA countries, highlighting the importance of democratic quality for environmental preservation. The insignificant value of spatial lagged variable of democratic quality (W*DQL) demonstrate that democratic quality of a country has not any impact on ecological footprint of bordering country. Finally, the estimated results depict that financial development is not appropriate for ecological footprint in BRI countries. It may be argued that financial development encourages the development of infrastructure and manufacturing activities and industry in BRI countries is heavily relying on fossil fuels for energy production which is spoiling the environment. Additionally, the negative relation of spatial lagged variable highlights that financial development is helpful to preserve the environment in the neighboring countries. As industrial expansion is observed in a region then labor starts to immigrate in that country due to job creation. The findings of the study are in line with findings of Samreen and Majeed [56], which explored the relation between CO2 emission and financial development.

## 6. Conclusions

This article is an attempt to investigate the spatial impact of ecological footprint and its affecting determinants in BRI participating economies. There are numerous studies analyzed the potential determinants of ECF but there is hardly any study that examined the spatial dependence of ecological footprint and productive capacities as a potential determinant of ecological footprint. It is a debate starting study exploring the spatial effects of ecological footprint. The empirical outcomes of the study reveal the significant spatial dependence in endogenous and exogenous variables. In simpler words, ecological footprint and economic activities in a country has the potential to affect the environment in neighbor country in a significant way. It is of great importance for policy makers to keep in view the consequences of a devised policy for local economy as well as for neighboring country.

The findings of this study highlight that many economic activities have impact on the country and environment of bordering country. It is possible that a factor affecting positively on a country’s environment may deteriorate the environment in neighboring country. For example, per capita GDP and financial development deteriorate the environment in a country while they have less detrimental impact on environment for a neighboring country. The green investment is the only factor which contributes to preserve the environment in the home country but it plays a positive role to improve the environment in the neighboring country. Even though it has a little contribution for environmental sustainability in BRI countries but a proper policy design may expand its effectiveness. The industries using green technology or pro-environment technology may be encouraged through tax rebates and subsidies etc.

The article "The usage of spatial econometric approach to explore the determinants of ecological footprint in BRI countries" was retracted in 2024. Reasons: compromised peer review; unreliable results or conclusions; concerns about the data; concerns about the peer review.

Moreover, it is also found that high democratic quality decreases the environmental challenges. The policies focusing to improve the judicial system, protection of human rights, and free media can reduce the environmental issues because they provide awareness to people regarding benefits of cleaner environment so people demand the rules and regulations to protect the environment. It also should keep in view that economic sanctions on the country decrease the priority of environmental protection and creates environmental issues [57]. The countries may design the policies where democracy may be practiced without any constraints. The public oriented governments care about citizens and their health so such policies are established by democratic governments which are environmental friendly.

The findings of the study have important academic and practical implications. The study contributes to the academic field through expansion of our understanding of the spatial impact of ecological footprints. Research on the spatial impact of ecological footprints in BRI countries may involve the development of innovative methodologies and analytical frameworks. This can enhance our ability to assess and quantify ecological footprints, understand their spatial patterns, and identify potential interventions for sustainable development. Moreover, the spatial impact of ecological footprints requires interdisciplinary research collaboration. Scholars from various fields like environmental sciences, geography, economics, and urban planning may collaborate to combat the environmental challenges of BRI countries.

The practical implications of the study may be policy formulation, regional cooperation and identification of most vulnerable areas of the region. The spatial analysis of ecological footprints may be used to identify the regions which require specific environmental protection measures and resource management strategies. Decision makers can use this information to identify areas with high environmental vulnerability and incorporate environmental considerations into infrastructure projects. In addition, the importance of international collaboration and knowledge sharing among BRI countries is highlighted. Various organizations can collaborate to exchange best practices, share environmental management techniques, and foster joint efforts for ecological conservation and sustainable development.

The article "The usage of spatial econometric approach to explore the determinants of ecological footprint in BRI countries" was retracted in 2024. Reasons: compromised peer review; unreliable results or conclusions; concerns about the data; concerns about the peer review.

The following policy recommendations can be made to reduce ecological footprint in BRI countries: there is need to invest more in green technology to reduce their dependence on natural resources. This investment may be for development of renewable energy sources such as solar, wind, and hydro power. This will not only reduce the ecological footprint but also improve the overall health of the public by reducing pollution. BRI countries should focus to increase their productive capacities for environmental preservation. This can be achieved through quality education and training of the workforce, and investment in research and development. Democratic quality ensures that policies related to the environment are implemented effectively. This can be achieved by promoting transparency, accountability, and citizen participation in decision-making processes. Given the spatial dependence of ecological footprint, BRI countries should promote regional cooperation to reduce the overall ecological footprint. This can be achieved through joint policies on environmental protection and sharing of best practices.

It should be emphasized that this research represents a first attempt to investigate the regional environmental quality-influencing components using a spatial econometric methodology. However, future research must use additional spatial econometric methods, such as regionally weighted regression and dynamic spatial panel data models. We propose extending the study by including other nations and years in the analysis. We conclude by recommending further research into how other significant factors, such as agricultural policies, R&D, transportation systems, and the variety of renewable energy sources, affect environmental quality.
